The article "Discussion on Health Service System of Mobile Medical Institutions Based on Internet of Things and Cloud Computing" was retracted in 2023. Reason: concerns about the peer review.

# Discussion on Health Service System of Mobile Medical Institutions Based on Internet of Things and Cloud Computing

**DOI:** 10.1155/2022/5235349

**Published:** 2022-01-07

**Authors:** Jinzhou Tang

**Affiliations:** School of Health Management, Xi'an Medical University, Xi'an 710021, Shaanxi, China

## Abstract

Because modern human beings pay more and more attention to physical health, and there are many problems in the traditional medical service system, human beings have a higher and higher voice for the new medical model. At present, there are many researches on the application of modern science and technology to put forward solutions to medical development, but they generally pay attention to some details and ignore the construction of the whole medical service system. In order to solve the problems of low efficiency of the traditional medical model, difficult communication between doctors and patients, unreasonable allocation of medical resources, and so on, this article proposes establishing a perfect medical and health service system. First, the correlation functions are used, such as cosine correlation, to calculate the correlation of various medical products, and then the correlation measurement methods of cloud computing and the Internet of Things are used to realize the network connection of smart medical equipment, efficiently store, calculate and analyze health data, and realize online outpatient services, health file management, data analysis, and other functions. Then, the energy consumption formula of the wireless transceiver was used to reduce the resource loss in the operation of the system. Then, we use the questionnaire to understand the current situation of mobile medical and put forward improvement suggestions. This article also scores the performance of the system. The experimental results show that the performance rating of traditional medical institutions is B, while the model rating of mobile medical institutions is a, and the efficiency is optimized by 4.42%.

## 1. Introduction

### 1.1. Background

In recent years, with the popularization and expansion of mobile smart devices and global mobile communication networks, the Internet of Things technology has been spawned, which is based on the Internet and extends the user side to between things. With the gradual increase in the business volume of the Internet of Things, a large amount of information exchange and communication has increased the demand for data storage, analysis, and computing capabilities, and cloud computing technology has emerged. Various mobile applications and services based on the Internet of Things and cloud computing have emerged. Many “ready-to-use” services have a lasting impact on people's lives. Application in the medical field can greatly improve the quality of services, expand the scope of services, and solve some of them [1, 2]. The problem of uneven distribution of medical resources has created a new medical method of “mobile medical.” Today's mobile medical institutions have implemented mobile application solutions such as wireless ward rounds, network calls, remote outpatient clinics, and mobile nursing services [3, 4]. Mobile technology can optimize patient consultation procedures such as inpatient registration, dispensing, sampling, surgery, and discharge. At the same time, it can benefit patients and healthcare professionals. Therefore, with the continuous development of mobile technology, users are increasingly demanding new medical service systems.

The article "Discussion on Health Service System of Mobile Medical Institutions Based on Internet of Things and Cloud Computing" was retracted in 2023. Reason: concerns about the peer review.

### 1.2. Significance

At present, the application of mobile medical services mainly focuses on providing services for medical staff and improving the efficiency of medical operations while ignoring personal tracking, electronic medical record management, etc. The health service system is not yet perfect. In this regard, this article proposes research on the medical and health service system of mobile medical institutions based on the Internet of Things and cloud computing [5]. Through the research of this article, a set of mobile medical and service systems based on mobile smart terminal equipment has been designed, which integrates various mobile medical data to achieve a more friendly service. There is a certain guiding significance.

The health service system is divided into three levels of management. The first layer is the community basic medical system, the second layer is the community general clinic, and the third layer is the urban comprehensive hospital. Community clinics provide the most basic healthcare services 24 hours a day. If necessary, doctors will transfer patients to the upper-level hospital. Such a system has played an important role for a long time and was once advertised by the British as “the most complete medical service system in the West.” The health service system of mobile medical institutions based on the Internet of Things and cloud computing can make today's health service system more scientific. Combining the transmission efficiency of the Internet of Things and the processing power of cloud computing can make the health service system have high efficiency and high data processing capabilities.

### 1.3. Related Work

With the progress of society, more and more people have conducted research on mobile medical institutions. Xa et al. defined cloud computing as a model that can realize ubiquitous, convenient, and on-demand network access and sharing of configurable computing resource pools. Their purpose was to develop and verify a tool to determine the determinants that affect the use of cloud computing. The factors include the attitude toward using cloud computing services (CCS), perceived privacy/security, perceived behavior control, the intention to use cloud computing services (CCS), and subjective norms. This research focuses not only on subjective factors but also on objective factors such as hardware facilities and other insufficient attention [6]. Huo et al. believed that while the computing efficiency of the industrial Internet of Things system is greatly improved, privacy issues may seriously damage the interests of users. They summarized the privacy issues in the industrial Internet of Things system and provided privacy when using software to define networks and blockchains. However, this solution can only solve network problems and has little effect on the physical level [7]. Yu et al. wanted to explore unique urban development models through new technologies such as the Internet of Things, cloud computing, and 4G and introduced successful experiences into all walks. However, building a smart city is a complex issue that requires multiple considerations of human factors and not just through technical means [8]. Avula believed that it was necessary to redesign the medical system to meet the needs of the people and quickly solved many complex problems in a shorter time and at a lower cost. He focused on the possibility of cloud computing technology in the medical field but only stayed at the theoretical research with no actual investigation [9]. Jeong et al. described the medical image information system for medical image sharing and used cloud services for the external interface of the system. They adjusted the connection of the device with PACS and smart devices and synchronized the data of the image application service based on cloud computing services. The research is a specific application case of the Internet of Things and cloud computing in mobile medical institutions, but it requires a lot of infrastructure investment, and small and medium medical institutions cannot achieve this effect [10]. Li et al. proposed two secure and efficient dynamic searchable symmetric encryption (SEDSSE) schemes for medical cloud data: using secure k-nearest neighbor (kNN) and attribute-based encryption (ABE) technology to construct a dynamic searchable symmetric encryption scheme; these two security attributes are crucial and extremely challenging in the field of dynamic searchable symmetric encryption. However, the problem of key sharing has not been solved yet, so that most people do not have the right to view information [11, 12]. Cao et al. believed that in the process of extensive deployment of the intelligent medical system, with the rapid development of medical equipment and the continuous increase of the number of medical equipment, it will become extremely difficult to plan or manage large-scale medical Internet of Things systems on the traditional single cloud platform. Various technologies should merge to reduce workload and provide medical data storage and backup mechanisms. However, medical service systems are rarely regular, and the work of merging similar items is not easy, but overinstitutionalized drawbacks will appear [13].

The article "Discussion on Health Service System of Mobile Medical Institutions Based on Internet of Things and Cloud Computing" was retracted in 2023. Reason: concerns about the peer review.

### 1.4. Innovation

The main innovations of the research content of this article are as follows. (1) Based on the development and deployment of the application platform, this article selects a mature and technologically advanced cloud service platform and makes full use of distributed database technology and distributed computing technology to realize data distributed storage. (2) Based on the analysis of the development status of Internet and cloud computing applications in the medical industry, we will boldly combine mobile information technology, apply our advantages to the field of medical services, and propose a mobile medical institution service system based on Internet of Things and cloud computing. (3) Pay attention to the current imbalance in the development of mobile medical institutions, focus on providing mobile medical solutions for vulnerable service institutions, shape a new industry service model, and realize the rational allocation of medical resources.

## 2. Methods of Mobile Medical Service System

### 2.1. Relevance Measurement of Cloud Computing

Many recommended algorithms use item correlation, and there are three most commonly used measurement methods: cosine similarity, adjusted cosine similarity, and correlation similarity [14].

Cosine correlation: cosine similarity measures the similarity between two vectors by calculating the cosine of the angle between them. It is widely used in calculating document similarity. The i_th_column of the user evaluation matrix, that is, the score vector of item *i*, is denoted as *r*_*i*_; the *j*_th_column, the score vector of item *j*, is denoted as *r*_*j*_; the set of users who have purchased item *i*and item *j*at the same time is *U*_*i*_, The correlation *W*_*ij*_between item *i*and item *j*can be measured by the angle between the vectors as follows:

(1) $$\begin{array}{c} W_{ij}=\cos\left(r,i,r,j\right)\\ =\frac{r,i\cdot r,j}{\left\|r,i\right\|\cdot \left\|r,j\right\|}\\ =\frac{\sum_{u\in U_{ij}}r_{ui}r_{uj}}{\sqrt{\sum_{u\in U_{i}}r_{ui}^{2}\sum_{u\in U_{j}}r_{uj}^{2}}}. \end{array}$$

Modified cosine correlation: the purpose of correcting the cosine similarity is to solve the cosine similarity that only considers the similarity in the direction of the vector dimension and does not consider the difference in the dimensions of each dimension. Therefore, when calculating the similarity, a correction operation of subtracting the mean value of each dimension will be performed. This method improves the cosine correlation without considering the insufficiency of different users' different scoring habits (high or low). It is calculated as follows:

(2) $$\begin{array}{c} W_{ij}=\frac{\sum_{u\in U_{ij}}\left(r_{ui}-r_{u}\right)\left(r_{uj}-r_{u}\right)}{\sqrt{\sum_{u\in U_{ij}}{\left(r_{ui}-r_{u}\right)}^{2}\sum_{u\in U_{ij}}{\left(r_{uj}-r_{u}\right)}^{2}}}. \end{array}$$

Correlation is also known as Pearson correlation. Correlation mainly considers a linear correlation, which is defined as the quotient of the covariance and standard deviation between two variables and is widely used to measure the degree of correlation between two variables. Correlation is the average score formula (3) of a single item and the average score formula (4) for calculating Pearson's correlation when calculating the item relevance.

(3) $$\begin{array}{c} W_{ij}=\frac{\sum_{u\text{Î}U_{ij}}\left(r_{ui}-r_{i}\right)\left(r_{uj}-r_{j}\right)}{\sqrt{\sum_{u\text{Î}U_{ij}}{\left(r_{ui}-r_{i}\right)}^{2}\sum_{u\text{Î}U_{ij}}{\left(r_{uj}-r_{j}\right)}^{2}}}, \end{array}$$

(4) $$\begin{array}{c} W_{uv}=\frac{\sum_{u\in I_{uv}}\left(r_{ui}-r_{u}\right)\left(r_{vi}-r_{v}\right)}{\sqrt{\sum_{u\in I_{uv}}{\left(r_{ui}-r_{u}\right)}^{2}\sum_{u\in I_{uv}}{\left(r_{vi}-r_{v}\right)}^{2}}}. \end{array}$$

It is generally believed that diversity is the opposite of correlation [15]. In the actual situation, recommending a group of similar items to users takes a lot of time to traverse the complete collection of items. If the similarity between items *j*and *i*is represented by *W*_*ij*_, where *W*_*ij*_∈ [0,1], *L*(*u*)is the list of items recommended by the system for user U, so the diversity of *L*(*u*)can be expressed by the following formula:

(5) $$\begin{array}{c} \text{diversity}=\frac{\sum_{i,j\in L\left(u\right),i\neq j}W_{ij}}{1/2\left|L\left(u\right)\right|\left(\left|L\left(u\right)\right|-1\right)}. \end{array}$$

When considering the list of recommended items of all users, the overall diversity should be averaged [16], and the following formula can be used:

(6) $$\begin{array}{c} \text{diversity}=\frac{1}{\left|U\right|}\sum_{u\in U}\text{Diversity}\left(L\left(u\right)\right). \end{array}$$

In the actual situation, the prediction accuracy of the recommendation algorithm will increase as the number of items increases and the additional calculations account for a small proportion of the total and can be ignored, but the introduction of the user list can increase the coverage, optimize resource allocation, and improve user satisfaction. [17]. It is generally believed that the coverage rate (Coverage) describes the share of items that can be recommended by the recommendation system. Simply put, it is the percentage of all items that can be recommended by the recommendation system. This formula can meet the docking of user and business information, achieve the accurate matching, and reduce resource waste. In formula (7), U is the user set, *L*(*u*)is the recommended item, and *G*is the set of all items. From a commercial point of view, the higher the coverage rate is, the more products we recommend to users. We can recommend the most in-demand medical products to users, which may result in higher user satisfaction and adequate and reasonable allocation of medical resources [18].

(7) $$\begin{array}{c} \text{coverage}=\frac{\left|U_{u\in U}L\left(U\right)\right|}{\left|G\right|}. \end{array}$$

The above is a recommendation algorithm based on item relevance and diversity, and the main idea of a content-based recommendation algorithm is to identify the common characteristics and attributes of items that have been given higher ratings by users and then identify those that have the same attributes as the item recommend new items to users [19]. The information containing the properties of item *j*is generally recorded in the form of the feature vector *x*_*j*_. User u's preference feature vector *x*_*u*_generally needs to be obtained from the user's rated item subset *L*(*u*). After the user's preference vector *x*_*u*_is obtained, it can be found that those new items whose feature vector *x*_*j*_is similar to *x*_*u*_are recommended to users [20].

(8) $$\begin{array}{c} X_{u}=\sum_{j\in L_{u}}r_{uj}x_{j}. \end{array}$$

The *U*_ser_*CF*algorithm predicts the user's rating *r*_*uj*_of item *j*using some users' ratings of item *j*similar to user *u*and uses *W*_*uv*_to represent the similarity between two users. We denote such a group of neighbors as *N*(*u*)[21]. Then, *r*_*ui*_can be estimated by averaging the scores of these neighbors on *j*.

(9) $$\begin{array}{c} {\text{r}}_{uj}=\frac{1}{\left|N_{j}\left(u\right)\right|}\sum_{v\in N_{j}\left(u\right)}r_{vj}. \end{array}$$

However, this formula still has a problem. It does not take into account the fact that each user has different evaluation standards and levels for items. The following formula gives a new method of score prediction [22]:

(10) $$\begin{array}{c} r_{uj}=h^{-1}\left(\frac{\sum_{v\in N_{j}\left(u\right)}w_{uv}h\left(r_{vj}\right)}{\sum_{v\in N_{j}\left(u\right)}\left|w_{uv}\right|}\right). \end{array}$$

*h*(*rvj*)in the formula represents the relative rating considering the average rating level of user *v*and h^−1^is the inverse function of *h*. For further explanation, see the following formula:

(11) $$\begin{array}{c} h\left(r_{uj}\right)=r_{uj}-r_{u}. \end{array}$$

If *W*_*ij*_is the similarity between items *i*and *j*and *L*(*u*)is the number of items that the user has rated, then the user's rating prediction for item *i*can be calculated by the weighted average of the ratings of all items in user u's item list *N*_*ui*_. Formula (12) is obtained. In the same way, formula (13) can be used for predictive scoring considering differences in personal scoring standards.

(12) $$\begin{array}{c} r_{ui}=\frac{\sum_{j\in L\left(u\right)}w_{ij}r_{ui}}{\sum_{j\in L\left(u\right)}\left|w_{ij}\right|}, \end{array}$$

(13) $$\begin{array}{c} r_{u\text{i}}=h^{-1}\left(\frac{\sum_{v\in L\left(u\right)}w_{ij}h\left(r_{uj}\right)}{\sum_{v\in L\left(u\right)}\left|w_{ij}\right|}\right). \end{array}$$

There is a distance threshold *d*_0_for communication between nodes that consume energy for wireless transmission between items and its value is determined by the external environment [23]. When the distance between the sending node and the receiving node is less than *d*_0_, the energy consumed to send data is proportional to the square of the distance [24]; it can be seen that the energy *E*consumption required to transmit bit information when the distance between nodes is *d*is as follows:

(14) $$\begin{array}{c} \text{E}=\left\{\begin{array}{cc} \text{kEelec}+{\text{kefd}}^{2}, & d<d0,\\ \text{kEelec}+{\text{kempd}}^{4}, & d>d0. \end{array}\right. \end{array}$$

Eelecrepresents the energy consumed by the wireless transceiver circuit; efd2and empd4represent the energy consumed by the signal amplifier to transmit each bit of data; *k*represents the length of the data packet; *d*represents the distance between the nodes. The energy consumption *E*_*r*_of the received signal and the formula considering the energy consumption of data fusion are as follows [25]:

(15) $$\begin{array}{c} Er=\text{kEelec,}\\ Er=k\left(\text{Eelec}+\text{Edf}\right). \end{array}$$

Although cloud computing and the Internet of Things are advanced science and technology, their basic application principles in the medical field are as follows. The main roles are only users (patients) and doctors, and the main medium is smart devices that can be combined through the network, supplemented by the service platform, solve practical problems, and improve efficiency for both parties [26, 27]. The basic schematic diagram is shown in Figure 1.

The article "Discussion on Health Service System of Mobile Medical Institutions Based on Internet of Things and Cloud Computing" was retracted in 2023. Reason: concerns about the peer review.

### 2.2. The Performance Evaluation Model of the Mobile Medical Institution Model

Compared with the traditional service model, the biggest difference of the mobile medical institution model is that the service process is realized by using the Internet of Things technology and a virtual cloud computing platform. Using the Internet of Things and cloud computing, it is possible to integrate the management and planning of the mobile medical institution model, resource supply and allocation, performance evaluation, etc., to build a systematic and holistic comprehensive system, and to easily integrate the medical information, which is passed to the hands of every citizen, realizing the full coverage of medical services in different regions and urban and rural areas [28, 29]. Therefore, to evaluate the performance of the mobile medical institution model, it is necessary to discuss the three aspects of service model innovation, service process reengineering, and public interest realization [19]. This article draws up initial performance evaluation indicators. The weighted average score refers to the average score calculated by multiplying each score by its weight ratio. Medical assessment scores can be set, and then, weights are set according to the contribution of each person's work, and the weighted average is used to reasonably evaluate the distribution performance. According to the structure of the construction and operation process of the cloud computing platform of the mobile medical institution, the first-level indicators of performance evaluation are constructed: (1) whether the mobile medical institution model is constructed in accordance with a reasonable plan; (2) whether the mobile medical institution model is operating in accordance with reasonable design requirements.

The construction process and operation process of the mobile medical institution model are subdivided, and six secondary indicators have been constructed: (1.1) whether the project management is normal; (1.2) whether the plan for model construction is implemented; (1.3) whether the process of managing nongovernmental organizations and enterprises participating in the construction of the model is carried out; (2.1) whether the platform is fully prepared for operation; (2.2) whether the management process of the model is effectively controlled; (2.3) whether the medical public service management planning process is effectively controlled and a quantifiable evaluation for each secondary index is established. Each of the five tertiary indicators is used to quantify and evaluate the construction process and operation process of the mobile medical institution model.

The article "Discussion on Health Service System of Mobile Medical Institutions Based on Internet of Things and Cloud Computing" was retracted in 2023. Reason: concerns about the peer review.

The relevance of each three-level indicator is assessed and scored. The classification of each level is based on the content of the hospital assessment and is divided into excellent, qualified, basic qualified, and unqualified according to the degree of completion of the work content. The scoring rules are as follows:10 points, requirements are fully implemented; 8 points, more than 3/4 requirements are implemented; 6 points, some requirements are implemented; 4 points, most requirements are not implemented, 0 points, there is no progress at all. According to the scoring of the third-level indicators, the implementation of the second-level indicators is calculated, and the calculation formula is as follows:

(16) $$\begin{array}{c} e\text{x}=\sum \frac{\text{ three}-\text{level indicator score}}{\text{ the highest possible score for the three}-\text{level indicator}}\left[\%\right]. \end{array}$$

Among them, *x*refers to each secondary index. According to the scores of the second-level indicators, the implementation of the first-level indicators can be calculated as follows:

(17) $$\begin{array}{c} e_{1}\%=\frac{e1.1+e1.2+e1.3}{3}\left[\%\right],\\ e_{2}\%=\frac{e2.1+e2.2+e2.3}{3}\left[\%\right],\\ e_{\text{overall}}\%=\frac{e1.1+e1.2+e1.3+e2.1+e2.2+e2.3}{3+3}\left[\%\right]. \end{array}$$

Among them, **e**_1_reflects the implementation of the mobile medical institution model during the construction process; **e**_2_reflects the implementation during the operation process; **e**_overall_reflects the implementation of the entire system from construction to operation. According to the scores of **e**_1_, **e**_2_, and **e**_overall_, the construction and operation process of the mobile medical institution model can be graded [30]. See Table 1for grading standards.

When the level is A, it means that there is basically no problem in the construction and operation of the mobile medical institution model, and the relevant departments can correct the related problems by themselves. When the grade is B, it indicates that there are certain problems in the construction and operation of the mobile medical institution model. The government department can rectify the related problems and then report to the performance evaluation department for review. When the level is C, it indicates that there are serious problems in the construction and operation of the mobile medical institution model. It should be reported to the superior authority immediately, and the rectification should be carried out under the supervision of the superior agency. After the rectification is completed, an application for a new performance evaluation should be applied.

The article "Discussion on Health Service System of Mobile Medical Institutions Based on Internet of Things and Cloud Computing" was retracted in 2023. Reason: concerns about the peer review.

### 2.3. Health Service System Architecture Diagram Design

This article selects Android and iOS devices, such as mobile devices, and sends real-time requests to the back-end server via HTTP. According to the user type and request type, the back-end service program makes the first evaluation, physical sign recording, patient browsing, and other operations according to the response type and stores them in the corresponding database. Do the corresponding data storage and data echo operations [15]? Business logic analysis and functional modeling for the system are conducted. The complete use case diagram includes the relationship between use cases, actors, and the system, which can effectively express a complete function provided or defined in the system and be perceived by users. The medical service system based on mobile smart terminals aims at medical service. The system is used to process, collect, and store patient information and diagnose diseases [31, 32]. The service system modeling is shown in Figure 2.

With the development of science and technology, mobile medicine plays an important role in clinical diagnosis, scientific research, and education [33]. How to effectively display a large amount of medical information on a limited number of mobile smart devices is a question worth considering. However, due to the resource limitations of mobile smart devices, mobile smart devices cannot handle complex tasks for a long time, like desktop systems. Therefore, this article proposes a threshold-based level set segmentation method for data segmentation under multi-threaded conditions.

## 3. Mobile Medical Service System Development and Achievement Analysis

### 3.1. The Public's Willingness to Adopt Mobile Healthcare

The mobile medical market in my country started late because of the slow process of informatization promotion, the low penetration rate of smartphones, the large and widespread population, and the imperfect medical system [34]. However, with the development of mobile technology becoming more and more mature and the popularization of smart terminals, China's mobile medical market has begun to sprout and emerge on a large scale. The experiment first analyzes the influencing factors of the people's willingness to use mobile medical applications so that the government can improve mobile medical according to the needs of the public, better realize the interaction between the government, enterprises, and the public, and play the role of mobile medical [35]. The questionnaire surveyed the medical needs of doctors and patients so as to realize the matching of needs and better optimize medical resources. The theme of the article is to build a medical exchange platform. First, study the development status of domestic mobile medical care. Taking Nanchang Maternity and Child Health Hospital as an example, the amount of medical payment and the number of payments in different ways are shown in Figure 3.

The article "Discussion on Health Service System of Mobile Medical Institutions Based on Internet of Things and Cloud Computing" was retracted in 2023. Reason: concerns about the peer review.

This shows that while the volume and number of online transactions increase, the market share of autonomous transaction machines is declining, and other forms of transactions, including traditional over-the-counter cash payments, are also being affected. To some extent, the number of transactions has dropped significantly.

Subsequently, the influencing factors of mobile healthcare were formally investigated. This article is designed after consulting related literature. Many experts and scholars at home and abroad have conducted research on this. The data is true and effective, which can guide article design very well, integrate various mobile medical data, and achieve more friendly services. At the same time, the survey questionnaire was distributed online and offline, and the questionnaire star was used online for questionnaire editing; offline questionnaires were distributed in universities, office buildings, hospital waiting rooms ,and other places. A total of 300 questionnaires were distributed online and offline. The questionnaire of the article is a one-to-one collection of data, the data are true and effective, and the degree of feasibility is extremely high. The data we collect is true and valid, and there is no invalid data. Among the valid samples in this questionnaire survey, the gender ratio is similar, with males accounting for 53% and females accounting for 47%. Young people aged 21–30 years old accounted for 58.3%, followed by people aged 31–40 years old accounting for 16%. In terms of education level, 77.3% of the population has a bachelor's degree or above, of which 20.3% have a master's degree or above and 57% have a bachelor's degree, indicating that the respondents generally have a higher degree of education. The respondents with a college degree accounted for 12% and a high school degree or below accounted for 11%. The young adults in the sample we selected came from other age groups. Their statements can guide the needs of other age groups. The popularity of the results is beyond doubt. See Table 2for the details of the respondents.

Through the analysis of the collected 300 valid questionnaires, descriptive statistics and correlation analysis methods are used to test the hypotheses proposed in the previous article. Based on the data of 300 surveys, we carried out the descriptive analysis and correlation tests and found that the survey results showed the needs of users very well, with advantages such as perceived usefulness, perceived ease of use, compatibility, social influence, and personal innovation can better know the upgrade and optimization of mobile medical. The results show that among a large number of influencing factors, perceived usefulness, perceived ease of use, compatibility, social influence, personal innovation, and willingness to adopt mobile medicine are significantly positively correlated. The correlation analysis coefficients are shown in Table 3.

The article "Discussion on Health Service System of Mobile Medical Institutions Based on Internet of Things and Cloud Computing" was retracted in 2023. Reason: concerns about the peer review.

### 3.2. Analysis of the Use of Mobile Medical Institutions

According to the survey results, with the advancement of national medical progress, mobile medical has developed rapidly. Thanks to the era of knowledge payment and the liberalization of medical e-commerce policies, the market scale of the mobile medical industry has grown rapidly, reaching 23.14 billion yuan in 2017, and the scale of the mobile medical market has reached 53.96 billion yuan in 2020. The scale of the medical market reached 53.96 billion yuan, and the growth is shown in Figure 4.

The questionnaire survey data indicated that patients hope to monitor their own health, medical history, and drug records through mobile medical services in the future, communicate with doctors better and more conveniently, and even realize remote monitoring of doctors. Doctors hope that mobile medical can help them increase real-time communication with patients, improve the quality of consultations, and optimize internal processes. The feedback from the questionnaire also showed that among the needs of doctor users, the expected data that have significantly changed from the current status also include communication with suppliers. The current needs of patients are covered by the needs they want to meet, and the two data can be directly synchronized. The demand situation of the patient and the doctor is shown in Figure 5.

As of September 2021, according to the data obtained from the survey, as a comprehensive health app, “Good Doctor Online” has been downloaded more than 180 million times. However, a more professional content system that can provide core medical services is relatively lacking. Mobile in the future medical developers has great prospects in providing more professional medical services based on how to deeply understand the needs of patients. On the other hand, statistics on doctor users show that as of September 2021, Dingxiangyuan's “Medical Time” active user market coverage reached 41.5%, and the second and third software belonged to Xingshulin among these applications that doctors often use. It is obvious that patients do not use them often. This is because these two have different expertise and needs and doctors and patients are still in different systems. When communicating, the transparency and openness of all information are limited. In general, the number of downloads by patients and doctors can be a good measure of coverage, and data collection is easy, and market coverage can be clearly perceived. The detailed market coverage of each application is shown in Figure 6.

The article "Discussion on Health Service System of Mobile Medical Institutions Based on Internet of Things and Cloud Computing" was retracted in 2023. Reason: concerns about the peer review.

### 3.3. Function Demonstration Based on Cloud Computing and Internet of Things

General mobile medical apps adopt the following model. Third parties such as smart medical equipment and pharmaceutical factories provide medical data. The app uses these data to build a two-way communication bridge between users and doctors. Doctors make diagnosis decisions based on the feedback data, and users follow the service. Scores are made to form a closed loop, and data generated during communication, such as electronic medical records, will provide samples for the database. Big data is provided by everyone who uses the system, and it is the ultimate storage terminal that can connect to all data. The detailed operation process is shown in Figure 7.

According to the existing mobile medical ecosystem in the abovementioned market, the mobile medical organization designed in this article relies on hardware and software. The hardware adopts sensor terminal products. There are many types of sensor terminals. Mainstream and high-quality sensor terminals on the market are chosen and their communication interfaces are transformed to make them compatible with mobile health protection projects. The relevant specifications of the project are connected to the gateway terminal of this project to complete the overall function of the system. At present, terminal hardware is divided into household multiparameter terminals and portable measurement terminals (including exercise blood glucose meters, monitoring rings, antidrop Bluetooth headsets, wrist blood pressure monitors, wrist electrocardiographs, and ECG phones) [36]. The software adopts the cloud platform service system, and the mobile medical health service system based on the cloud platform is composed of business processing, user service, business management, system management, expert system, user, and other subsystems [37]. The software architecture diagram of the mobile health service system platform is shown in Figure 8.

The business processing subsystem provides remote diagnosis, treatment, and health consultation services. Hospital experts use the physiological indicators collected by the health terminal to make preliminary and follow-up diagnoses of user indicators, give doctors guidance, start a rescue, make diet and medical plans, recommend services, etc. There are many types of service products, such as SMS, voice, video, and access [38]. At the same time, we can also provide call center agent services. The business processing subsystem also provides emergency rescue services. In other words, the user can initiate a “one-key rescue” request through a dedicated button on the emergency rescue terminal. The system recognizes the user's identity according to the user's rescue terminal number, confirms it, and then sends a rescue request work order to the rescue system (ambulance or medical institution in a nearby hospital). The user service subsystem is located in the user service subsystem. Users can measure indicators and upload data to the business platform through health sensing terminals and health information gateways. Users can change and update their personal profile information and view location information and billing status. Users can also create medical advice, weekly and monthly reports, health information, health indicators, and other information [39].

The article "Discussion on Health Service System of Mobile Medical Institutions Based on Internet of Things and Cloud Computing" was retracted in 2023. Reason: concerns about the peer review.

With this system, the author simulated online consultation, commuting time, case acquisition, registration, payment, laboratory test receipt, insurance reimbursement, and multiple processes, which is shown in a scatter chart.  Figure 9shows the processing time of the seven processes in order from left to right, including online consultation, commuting time, case acquisition, registration and call, payment, test paper collection, and insurance reimbursement. It can be seen from Figure 9that the processing time of mobile medical treatment far exceeds that of traditional medical treatment in many aspects, and the efficiency is improved significantly.

The traditional medical model determines the performance based on the performance of the medical workers, and the mobile medical institution evaluates the performance based on the weighted average of the level of the hospital's assessment, which is fairer. According to the performance of the evaluation model of the traditional medical institution model proposed above, this system is evaluated, and the calculated scores are shown in Table 4.

According to the formula, the traditional medical institution score of **e**_1_is 88.20%, the mobile medical institution score is 93.81%, the traditional medical institution score of **e**_2_is 90.67%, and the mobile medical institution scores 93.89%. In the aggregate score **e**_overall_, the traditional medical institution scores 89.43%. Mobile medical institutions scored 93.85%.  Figure 10is obtained according to the scoring details.

The article "Discussion on Health Service System of Mobile Medical Institutions Based on Internet of Things and Cloud Computing" was retracted in 2023. Reason: concerns about the peer review.

Traditional medical institutions have **e**_overall_score of 89.43%, less than 90%, and a performance rating of B, while the mobile medical institution model proposed in this article has a score of 93.85% and a rating of A. In addition, the small scores are also higher than the traditional medical institution as a whole. It can be seen that the health service system is efficient and executable.

## 4. Discussion

This article first introduces technologies such as the Internet of Things and cloud computing, understands the research status of mobile medical institutions through previous literature reviews, and designs mobile medical institutions through experimental methods such as cloud computing correlation measurement and mobile medical institution performance evaluation models. The health service system, through the experimental method of the questionnaire survey, understands the current status and problems of the current mobile medical service system and proposes the author's suggestions accordingly, intending to perfect this system. This article conducted a questionnaire survey on the public's willingness to adopt mobile medical services and obtained more real first-hand data. However, limited by the author's personal ability, time, and funding, this research has some shortcomings. Opinions are for reference for follow-up research. (1) The study sample has limitations. The sample in this article mainly covers Nanchang, but the population and medical conditions of various regions in China are different, and there is no nationwide sampling. (2) This article is mainly based on cloud computing for the application of medical software for the Internet of Things; future scholars can consider research on users' willingness to adopt more new technologies such as artificial intelligence. (3) The deep integration of sensors and smartphones is promoted to eliminate the demand for a variety of complex and bulky medical devices.

## 5. Conclusions

Based on the use of hardware and software facilities, this article relies on cloud computing and Internet of Things technology to realize online outpatient services, health file management, data analysis, and other functions. Mobile medical software can meet the needs of patients seeking medical advice. Users can browse Internet information and communicate directly with doctors and experts. Through research, this article puts forward the following suggestions for the health service system of mobile medical institutions. Intelligent medical equipment to carry health monitoring and personal monitoring services for people living alone can be connected with the hospital system to collect health-related data to the greatest extent. The mobile medical service system uses various ready-made resources such as health sensor terminals, communication networks, medical and health institutions, and communication operators, which reduces the cost of building a cloud platform. To improve the mobile medical system, we must give full play to the government's advantages, improve the establishment of related systems, and strengthen publicity and promotion to let more people understand the mobile medical system. The design of mobile medical applications is optimized to ensure the security and user privacy of a large amount of health data.

The article "Discussion on Health Service System of Mobile Medical Institutions Based on Internet of Things and Cloud Computing" was retracted in 2023. Reason: concerns about the peer review.

## Figures and Tables

**Figure 1:** Basic principles of mobile healthcare.

**Figure 2:** Business analysis of the health service system of mobile medical institutions.

**Figure 3:** Statistics chart of the payment amount (ten thousand yuan) and the number of transactions by different payment methods.

**Figure 4:** 2015–2020 China's mobile medical (service) market status.

**Figure 5:** Patient-doctor's functional requirements for mobile medical institutions.

**Figure 6:** The number of patient app downloads, doctor app coverage.

**Figure 7:** Mobile medical ecosystem.

**Figure 8:** Software operation architecture diagram.

**Figure 9:** Scatter plot of processing time for different medical modes (minutes).

**Figure 10:** Performance score chart of the traditional medical model and mobile medical institution model.

**Table 1:** Grading standards.

Grade	Score	Illustration
A	*e* ≥ 90%	There is basically no problem in the construction and operation of the system
B	80%≤*e*<90%	There are certain problems in the construction and operation of the system
C	*e* ≤ 80%	There are serious problems in the construction and operation of the system

**Table 2:** Basic information of survey samples.

Variable	Type	Frequency	Percentage
Gender	Male	159	53.0
	Female	141	47.0
	Total	300	100.0

Age	Under 20	17	5.7
	21–30 years	175	58.3
	31–40 years	48	16.0
	41–50 years	38	12.7
	Above 50	22	7.3
	Total	300	100.0

Education	High school	32	10.7
	Junior college	36	12.0
	Undergraduate	171	57.0
	Master	58	19.3
	PhD and above	3	1.0
	Total	300	100.0

Income	3000 yuan and below	176	58.7
	3000–5000 yuan	83	27.7
	5000–8000 yuan	35	11.7
	8000 yuan and above	6	2.0
	Total	300	100.0

Profession	Student	169	56.3
	Civil servants	19	6.3
	Institutional personnel	15	5.0
	Enterprise personnel	45	15.0
	Individual/private owners	34	11.3
	Freelancer	5	1.7
	Unemployed	8	2.7
	Others	5	1.7
	Total	300	100.0

**Table 3:** Correlation coefficients between willingness to adopt and predictors.

		Optimism	Usefulness	Ease of use	Compatible	Resistance	Risk	Social	Innovation
Optimism	Correlation	1	0.619^∗∗^	0.561^∗∗^	0.460^∗∗^	−0.136^∗^	−0.06	0.441^∗∗^	0.556^∗∗^
	Significance	0.0	0.0	0.0	0.0	0.349	0.034	0.0	0.0

Usefulness	Correlation	0.475^∗∗^	1	0.620^∗∗^	0.624^∗∗^	−0.07	−0.018	0.383^∗∗^	0.401^∗∗^
	Significance	0.0		0.0	0.0	0.258	0.78	0.0	0.0

Ease of use	Correlation	0.621^∗∗^	0.561^∗∗^	1	0.529^∗∗^	−0.079	−0.032	0.479^∗∗^	0.370^∗∗^
	Significance	0.0	0.0		0.0	0.625	0.221	0.0	0.0

Compatible	Correlation	0.460^∗∗^	0.475^∗∗^	0.529^∗∗^	1	−0.158^∗^	−0.033	0.355^∗∗^	0.480^∗∗^
	Significance	0.0	0.0	0.0		0.014	0.61	0.0	0.0

Resistance	Correlation	−0.136^∗^	−0.073	−0.079	−0.158^∗^	1	0.245^∗∗^	−0.04	−0.247^∗∗^
	Significance	0.034	0.258	0.221	0.014		0	0.535	0.0

Risk	Correlation	−0.06	−0.017	−0.032	−0.033	0.245^∗∗^	1	0.042	−0.029
	Significance	0.349	0.78	0.625	0.61	0.0		0.613	0.557

Social	Correlation	0.456^∗∗^	0.401^∗∗^	0.481^∗∗^	0.356^∗∗^	−0.04	−0.029	1	0.237^∗∗^
	Significance	0.0	0.0	0.0	0.0	0.042	0.657		0.0

Innovation	Correlation	0.541^∗∗^	0.383^∗∗^	0.370^∗∗^	0.480^∗∗^	−0.251^∗∗^	0.535	0.236^∗∗^	1
	Significance	0.0	0.0	0.0	0.0	0.0	0.514	0.0	

∗∗Significantly correlated at the. 01 level (two-sided). ∗Significantly correlated at the 0.05 level (two-sided).

The article "Discussion on Health Service System of Mobile Medical Institutions Based on Internet of Things and Cloud Computing" was retracted in 2023. Reason: concerns about the peer review.

**Table 4:** Performance scoring table of the traditional medical model and mobile medical institution model.

Project	Existing medical model		Mobile medical service system	
	Average	Ideal highest	Average	Ideal highest
1.1. Is the project management normal	5.8	7	8.7	9
1.2. Has the construction plan been implemented	4.4	5	5.6	6
1.3. Whether to manage NGOs and businesses	7.5	8	6.4	7
2.1. Is the preparation before operation sufficient	5.8	6	8.7	9
2.2. Whether the management is effectively controlled	4.6	5	7.5	8
2.3. Whether the plan is effectively controlled	5	6	7.3	8

## Data Availability

The data that support the findings of this study are available from the corresponding author upon reasonable request.
